The article "Effectiveness of Insole Colour on Impact Loading and Lower-Limb Kinematics When Running at Preferred and Nonpreferred Speeds" was published in 2021. Journal: J Healthc Eng.

# Effectiveness of Insole Colour on Impact Loading and Lower-Limb Kinematics When Running at Preferred and Nonpreferred Speeds

**DOI:** 10.1155/2021/8947433

**Published:** 2021-12-01

**Authors:** Yi Wang, Wing-Kai Lam, Lok-Yee Pak, Charis K.-W. Wong, Mohammad F. Tan, Aaron K.-L. Leung

**Affiliations:** ^1^Department of Physical Education, Renmin University of China, Beijing 100872, China; ^2^School of Life Science and Technology, Harbin Institute of Technology, Harbin 150001, China; ^3^Humanistic Olympic Studies Center, Renmin University of China, Beijing 100872, China; ^4^Li Ning Sports Science Research Center, Li Ning (China) Sports Goods Co. Ltd., Beijing 101111, China; ^5^Department of Kinesiology, Shenyang Sports University, Shenyang 110102, China; ^6^Department of Biomedical Engineering, The Hong Kong Polytechnic University, Hong Kong 999077, China

## Abstract

While colour of red can play a significant role in altering human perception and performances, little is known about its perceptual-motor effect on running mechanics. This study examined the effects of variations in insole colours on impact forces, ankle kinematics, and trial-to-trial reliability at various running speeds. Sixteen male recreational runners ran on instrumented treadmill at slow (90%), preferred (100%), and fast (110%) running speeds when wearing insoles in red, blue, and white colours. We used synchronized force platform and motion capturing system to measure ground reaction force, ankle sagittal and frontal kinematics, and movement variability. A two-way (colour x speed) ANOVA with repeated measures was performed with Bonferroni adjusted post hoc comparisons, with alpha set at 0.05. Data analyses indicated that participants demonstrated higher impact and maximum loading rate of ground reaction force, longer stride length, shorter contact time, and smaller touchdown ankle inversion as well as larger ankle sagittal range of motion (RoM), but smaller frontal RoM in fast speed as compared with preferred (*P* < 0.05) and slow speeds (*P* < 0.001). Although insole colour had minimal effect on mean values of any tested variables (*P* > 0.05), participants wearing red-coloured orthoses showed higher coefficient of variation values for maximum loading rate than wearing blue insoles (*P*=0.009). These results suggest that running at faster speed would lead to higher impact loading and altered lower-limb mechanics and that colour used on the tops of insoles influences the wearers' movement repeatability, with implications for use of foot insole in running.

## 1. Introduction

Running is a recreational sport to improve health and fitness as well as social influence. However, about 37–79% of the runners in a given year were reported to experience running-related injuries at lower extremity [1]. In general, lowering impact loading and improving rearfoot stability have been hypothesized to reduce the risk potentials [2–4]. Foot insoles (or refer to shoe orthosis/inserts) are commonly prescribed in sports community, as the insoles that contour foot plantar surface are often used to improve comfort [5], reduce impact loading [5, 6], and facilitate lower-limb mechanics and upper extremity performances [6, 7].

The article "Effectiveness of Insole Colour on Impact Loading and Lower-Limb Kinematics When Running at Preferred and Nonpreferred Speeds" was published in 2021. Journal: J Healthc Eng.

While most of the insole studies have predominantly investigated the effect of insole materials, hardness, or geometry in various sports [5–8], few studies have considered how the colour of insoles influences running performances [9]. Sportswear colour has been suggested to contribute to human perception, injury potential, and sport performances for its psychomotor influence [9–11]. Clinically, prefabricated insoles often use colours to denote specific material hardness for different populations and sports to increase the compliance of the patient wearing. It is reported that sharp colours (e.g., red and orange) induced higher perceived pain intensity than dark colours (e.g., black and grey), resulting in poorer performances [12]. Specifically, red colour is identified as the highest pain intensity in patients with osteoarthritis [13]. However, the opposite effect is evident in the context of sport domain and athlete population. Red colour has been suggested to correlate with positive feelings such as aggressiveness, power, and dominance [9, 11, 14] and can lead to better performances in various combat sport situations [11, 15–17]. Akin to insole study, participants wearing red would have impact on self-predicted performance [18], greater leg strength [19], and improved explosive motor performance [15], indicating a psychomotor influence. It is questionable if wearing red-coloured insoles may also enhance performance in noncombat environment.

A recent study examined the insole colour effect in a noncombat laboratory-based movement task [20], which had healthy basketball players performing drop landing from different heights in identical insoles with various colours of top-cover. Although the insoles were made of identical material and surface geometry, the participants wearing red insoles would induce better perception of forefoot and rearfoot cushioning and overall comfort as well as smaller plantarflexion moment than the white insoles. Given that the material and mechanical characteristics of the tested insoles should have been identical [20], it seems reasonable to conclude that the reported biomechanical differences were due to psychological and/or physiological factors associated with colour, even though the insoles used are not visible/perceivable by wearers during the sport activities [9]. Furthermore, researchers postulate that colour of an athlete's uniform influences their psychological functioning and thus leads to changes in sports performance [21]. Running performance is influenced by running economy which is significantly correlated with biomechanical variables [22]. There are researches lacking in the study of the influence of colour on running biomechanics. Considering the fact that running is a fundamental movement to any sports, there is a practical value in further understanding the effect of coloured insoles on running mechanics for large population in running community.

The article "Effectiveness of Insole Colour on Impact Loading and Lower-Limb Kinematics When Running at Preferred and Nonpreferred Speeds" was published in 2021. Journal: J Healthc Eng.

As noted, while running speed is associated with vertical ground reaction force, stride frequency, stride length, and ankle kinematics [23], executing a preferred running speed requires smaller effort and attention to maintain movement reliability/stability than a faster or slower nonpreferred speed [24]. Thus, the interplay effect between insole colour and running speed on gait parameters and movement reliability is questionable and might shed light on the underlying mechanism of the use of coloured insoles in running. Hence, the purpose of this study was to examine whether insole colour would influence spatial-temporal, impact loading, ankle kinematics, and trial-to-trial reliability when running at slow (90%), preferred (100%), and fast (110%) speeds. We hypothesized that red insoles would alter ankle mechanics and lower impact forces and trial-to-trial reliability [e.g., lower coefficient of variation (CV)] [16]. Such information would help coaches, sport scientists, and athletes in understanding the effectiveness of coloured insoles across different speeds.

## 2. Materials and Methods

### 2.1. Insole Colour Conditions

Three identical insoles with different top-surface colours (red, blue, and white) were built and all insoles had arch-support based on the specification of the off-the-shelf orthosis (sports arch-support series-Universal II, Dr. Kong Footwear Ltd, Hong Kong; Figure 1). To minimise the potential influence by shoe constructions, all insole conditions were fit and placed inside the identical neutral running shoe (Li Ning ARBM181, Beijing, China).

### 2.2. Participants

A priori power analysis indicated that a minimum number of 15 participants were required to obtain *α* = 0.05, effect size = 0.80 large, and power = 0.80. To avoid potential dropouts, we recruited sixteen male recreational runners (mean ± standard deviation: age = 25.2 ± 4.9 years, body height = 1.70 ± 2.31 m, body weight = 70.4 ± 4.1 kg) for this study. Only the participants with normal foot arch were included in this study, as they represented a broader population of recreational runners. Their arch index ranged between 0.21 and 0.28 based on the standard arch index method to categorize as normal arch [25]. Participants had no lower extremity injuries motor, cognitive disorders, and colour blindness in the past 6 months prior to the study. The colour blindness was checked using the Ishihara Colour Blindness test [20, 26]. The study was conducted in accordance with the Declaration of Helsinki and the procedure was approved by the Ethics Committee of Li Ning Sports Science Research Center (approval number: IRB-2017-BM016) on 10 September 2017.

The article "Effectiveness of Insole Colour on Impact Loading and Lower-Limb Kinematics When Running at Preferred and Nonpreferred Speeds" was published in 2021. Journal: J Healthc Eng.

### 2.3. Experimental Procedures

All participants included in this study were fully informed and debriefed forms were signed before and after the study, respectively. A debriefing form was necessary since the study objective was not fully disclosed in the informed consent to avoid bias associated with knowledge of colour manipulation, as previously reported [20]. To avoid any environmental changes that lead to biasness of colour perception, the same lighting was controlled in the biomechanical laboratory across participants [20].

Using a within-study design, participants were instructed to run with three coloured insoles (red, blue, and white) at slow (90%), preferred (100%), and fast (110%) speeds on the instrumented treadmill (Bertec Corp., Columbus, Ohio, USA). The running speed was selected in accordance with the previous study [8]. After anthropometric measurements were taken, participants were allowed to perform a 15-min self-administrative warm-up on the treadmill. The same experimenter placed reflective markers (diameter 14 mm) over the following landmarks (Figure 2): left and right ASIS and PSIS, medial and lateral femur epicondyles, medial and lateral malleolus, three calcaneus markers (posterior upper, lower, and lateral aspect of calcaneus), two foot tracking markers (medial side of first metatarsal head, upper side of second metatarsal head, and lateral side of fifth metatarsal head), and two rigid clusters of four markers that were attached onto the thigh and lower leg. The malleolus and femoral epicondyles markers were captured during static trials and then removed during running trials, as previously reported [8].

Participants were instructed to tighten their shoelaces as they would perform for endurance runs. Individual preferred speed was determined when the participants reported a comfortable running speed across the increase of treadmill speeds without seeing the exact speed, as previously described [8, 24]. This preferred speed (100%, 2.51 ± 0.40 m/s) was used to determine the slow (90%, 2.26 ± 0.36 m/s) and fast speed (110%, 2.77 ± 0.44 m/s) for this study.

The article "Effectiveness of Insole Colour on Impact Loading and Lower-Limb Kinematics When Running at Preferred and Nonpreferred Speeds" was published in 2021. Journal: J Healthc Eng.

Prior to each running condition, the participants were asked to gaze at the tested insole for 30 seconds to be reminded of which insole colour was being worn. Then, the participants ran for 1.5 minutes each condition and the last 10 consecutive steps were selected for further analysis [8]. Force plates (sampling at 1000 Hz) and 8-camera motion analysis system (sampling at 200 Hz) were synchronized to record ground reaction forces, spatial-temporal, and ankle kinematic information. To ensure the reliability of ground reaction force (GRF) data, the treadmill was calibrated and checked in accordance with standard procedure before data acquisition [27, 28]. A 5-min rest period was given for each speed and insole condition, as previously reported [28]. The order of insole and speed condition was randomly presented across participants.

### 2.4. Data Processing

All marker trajectories were identified and transferred into Visual3D software (C-Motion Inc., Ontario, Canada) to determine body segments and joint kinematic variables, as previously used [8, 28]. A spline interpolation was performed to fill any minor missing data using three frames before and after the missing data. The kinematics and GRF data were filtered using a fourth-order, zero phase lag, Butterworth low path digital filter at cut-off frequencies of 100 Hz and 50 Hz respectively, as previously reported [3, 8]. The stance phase was identified from initial contact to toe-off. The instant of initial foot-ground contact and toe-off were defined when the vertical GRF first went above and below 20 N, respectively [8, 28]. Peak impact and maximum loading rate of the vertical GRF, strike length, and ankle kinematics (i.e., sagittal and coronal touchdown angle and range of motion) were selected in this study as these variables were of direct relevance to study foot insole and running performance in accordance with previous studies [3, 8, 23, 28].

### 2.5. Statistical Analysis

The group mean and coefficient of variation (CV) were calculated from the last 10 consecutive running trials for statistical analyses (SPSS v22.0, Chicago, IL, USA). Initial Shapiro–Wilk tests validated that all data were normally distributed. When Mauchly's test assumption was violated, Greenhouse–Geisser's epsilon adjustment was used in all cases. The two-way (colour x speed) ANOVA with repeated measures were performed to determine if there was any significant interaction and main effect (*P*=0.05) for each variable. When any significant main effect was determined, the Bonferroni post hoc analyses were employed. Effect sizes (Cohen's *d*) were interpreted as follows: (i) small if 0.2 ≤ *d* < 0.5; (ii) medium if 0.5 ≤ *d* < 0.8; and (iii) large if *d* ≥ 0.8 [29].

The article "Effectiveness of Insole Colour on Impact Loading and Lower-Limb Kinematics When Running at Preferred and Nonpreferred Speeds" was published in 2021. Journal: J Healthc Eng.

## 3. Results

### 3.1. Effect of Insole Colour on Footwear Cushioning and Ankle Biomechanics

The ANOVA indicated the significant main effect of speed on impact loading, spatial-temporal, and ankle kinematics variables (*P* < 0.001), except ankle dorsiflexion at touchdown (Table 1). No significant main effects of colour and interaction were indicated. Participants with slow running speed exhibited significant lower peak impact forces (2.22 BW) than preferred (2.30 BW, *P* < 0.001, *d* = 0.31) and fast (2.35 BW, *P* < 0.001, *d* = 0.48) speeds and also lower maximum loading rate (93.06 BW/s) than preferred (101.35 BW/s, *P* < 0.001, *d* = 0.42) and fast (108.69 BW/s, *P* < 0.001, *d* = 0.67) speeds. In addition, participants running at preferred speed (2.22 BW) led to smaller peak impact force compared with the fast running speed (2.35 BW, *P*=0.012, *d* = 0.18).

For spatial-temporal parameters (Table 1), participants with slow running speed demonstrated larger contact time (0.29 s) than the preferred (0.28 s, *P* < 0.001, *d* = 0.73) and fast (0.26 s, *P* < 0.001, *d* = 1.25) speeds. However, the slow running condition showed smaller stride length (1.63 m) than preferred (1.78 m, *P* < 0.001, *d* = 0.91) and fast (1.94 m, *P* < 0.001, *d* = 1.68) running speed conditions. The preferred speed condition led to larger contact time (0.28 s, *P* < 0.001, *d* = 0.64) and smaller strike length (1.78 m, *P* < 0.001, *d* = 0.79) than the fast speed condition (contact time: 0.26 s; strike length: 1.94 m).

For ankle kinematics parameters (Table 1), participants with slow running speed demonstrated larger ankle inversion at touchdown (2.05°) than in fast running speed (1.67°, *P*=0.005, *d* = 0.36) and it had smaller angle sagittal RoM (29.71°) than preferred (30.76°, *P*=0.005, *d* = 0.33) and fast (31.50°, *P*=0.002, *d* = 0.59) speed conditions. Additionally, larger ankle frontal RoM was displayed in fast speed (10.34°) compared with slow (9.20°, *P* < 0.001, *d* = 1.01) and preferred (9.67°, *P*=0.022, *d* = 0.52) running speeds.

### 3.2. Effect of Insole Colour on Movement Variability

For movement variability variables (Table 2), the ANOVA indicated the significant main effect of colour on maximum loading rate (*P*=0.033) and main effect of speed on ankle sagittal RoM (*P*=0.038). Participants wearing red-colored insoles experienced higher CV values for maximum loading rate (14.08%) than wearing blue insoles (11.85%, *P*=0.009, *d* = 1.23). Participants with slow running speed demonstrated larger CV values for ankle sagittal RoM (8.06%) compared with the preferred (6.89%, *P*=0.027, *d* = 0.82) and fast (7.12%, *P*=0.045, *d* = 0.91) running speeds.

The article "Effectiveness of Insole Colour on Impact Loading and Lower-Limb Kinematics When Running at Preferred and Nonpreferred Speeds" was published in 2021. Journal: J Healthc Eng.

## 4. Discussion

While colour of red is often used to manipulate human perception, compliance of using insoles, and competitive sport performances [9–14], it is questionable whether red-coloured insoles would be beneficial [11, 14] or have deteriorated [12, 13] effect on daily activities such as walking and running that are fundamental to any sport movements. This study sought to examine if the insole colour would influence impact forces, joint kinematics, and its trial-to-trial reliability when running at slow (90%), preferred (100%), and fast (110%) speeds. When running at faster speeds, participants experienced higher impact loading, longer stride length, shorter contact time, and smaller touchdown ankle inversion as well as larger ankle sagittal RoM but smaller frontal RoM when compared with slower speeds. The higher GRF loading was associated with faster running speeds, which is mostly consistent with the previous literature [29]. The increased impact loading is hypothesized to impose a higher risk potential of running-related injuries [30]. A previous computational model study reported that higher knee contact forces were found when participants were walking/running at higher speeds [31]. Moreover, the high loading rate could be associated with longer stride length and/or higher step frequency at faster speeds. When running at faster speeds, smaller initial ankle inversion at touchdown could be related to smaller range of motion in frontal plane. The larger ankle sagittal but smaller frontal RoM could be attributed to the specific movement strategies adapted to various running speeds [32].

On the basis that visual perception and motor performance are intricately linked, red-coloured apparels might have outperformed in different combat sport contexts [11, 15–17]. Some previous studies also showed that wearing red may increase lower-leg strength [19] and enhance the force and velocity of motor output [14]. However, our results did not show any significant differences among red, blue, and white insoles for all tested variables in a noncompetitive running task. This is consistent with the previous sportswear colour study [18], which showed no actual soccer shooting accuracy and lower-leg kicking power among red, blue, and black bibs. However, this is not in line with the previous insole colour study on landing task [20], which showed that participants wearing red insoles would induce better cushioning perception and smaller ankle plantar flexion moment during landing when compared with the white-flat insoles. One possible explanation is that the influence of colour could be more effective when the participants are looking at the colour stimulus (e.g., opponent's outfit), rather than the insoles that are covered and unseen by the participants. Another explanation is that colour manipulation is in a different relation to the performers themselves when compared to their opponents [11]. Moreover, the movement task tested (running versus landing) would be one of the plausible explanations to cause the discrepancy of colour effect across the colour insole studies. More importantly, the influence and belief of colour could simply reflect culture and sport-specific associations [33], which explains contradictory findings across studies. While some studies reported that participants/teams wearing red outfits won more games than those wearing blue outfits in English Premier League [34], no relationship between wearing red uniforms and advantages can be found in Spanish League [15]. Importantly, one plausible explanation is the participant belief in the effectiveness of the colour manipulation in landing or running task. It has been reported that performance benefits of footwear/equipment can be maximized when one is confident with the proposed benefits of the worn footwear [35]. Future study should examine the efficiency and belief of insole colour in runners from different countries before a viable conclusion can be made.

The article "Effectiveness of Insole Colour on Impact Loading and Lower-Limb Kinematics When Running at Preferred and Nonpreferred Speeds" was published in 2021. Journal: J Healthc Eng.

Concerning the intertrial reliability, our results revealed that participants wearing red-coloured insoles experienced higher CV values for maximum loading rate than wearing blue insoles and that larger CV values for ankle sagittal RoM were found in slow speed than the other two faster running speeds. This is in line with the previous study, which indicated that wearing red jersey would be able to show higher CV values in participants in combat sports [19]. As the previous studies reported that lower intertrial variability during the early stance phase was related to the localised mechanical stress on a body in running [36], higher CVs found in red-coloured insoles might be related to the benefits of lowering injury risk.

When interpreting our results, some limitations should be considered. First, only male runners were recruited in this study. The current findings may not be generalizable to different gender and running levels. Females might have caused greater influence by the appearance of footwear in comparison to males, showing a larger discrimination between insole conditions. Second, we did not measure comfort perception variables. Comfort perception has sparked considerable interests to coaches and sports scientists, as better perceived comfort was related to lower incidence of sport injury [37], better running economy [38], and impact attenuation [39]. Future study may investigate if coloured insoles improve comfort, biomechanics, and performance in running.

The article "Effectiveness of Insole Colour on Impact Loading and Lower-Limb Kinematics When Running at Preferred and Nonpreferred Speeds" was published in 2021. Journal: J Healthc Eng.

## 5. Conclusions

Compared with slower speeds, running at higher speed led to higher impact loading, longer stride length, shorter contact time, smaller touchdown ankle inversion, and larger ankle sagittal RoM. Although the colour manipulation on sport insoles has no to minimal influence on actual impact loading, spatial-temporal, and ankle kinematics in recreational runners, participants wearing red-coloured insoles would lead to higher CV value for maximum loading rates. The significant findings in intertrial reliability could be insightful, with an implication for motor control strategy in the use of foot insole in running population.

## Figures and Tables

**Figure 1:** Three coloured insole conditions.

**Figure 2:** Markerset placement.

**Table 1:** Mean and SD of ground reaction force, spatiotemporal and joint angle variables by insole colour, and speed conditions.

Variables	Speed	Red	Blue	White	ANOVA (*P* value)			Post hoc
					Colour	Speed	Interaction	
Peak impact force (BW)	S	2.18 (0.28)	2.21 (0.26)	2.26 (0.31)	0.140	**<0.001** ^*∗*^	0.426	S < P, F; P < F
	P	2.25 (0.29)	2.32 (0.27)	2.33 (0.29)				
	F	2.34 (0.29)	2.33 (0.30)	2.38 (0.32)				

Max loading rate (BW/s)	S	91.22 (20.15)	92.65 (20.61)	95.31 (24.03)	0.285	**<0.001** ^*∗*^	0.774	S < P, F
	P	96.75 (23.17)	100.58 (23.75)	106.73 (25.46)				
	F	106.62 (28.67)	107.74 (27.23)	111.72 (30.34)				

Contact time (s)	S	0.30 (0.02)	0.29 (0.02)	0.29 (0.03)	0.556	**<0.001** ^*∗*^	0.177	S > P, F; P > F
	P	0.28 (0.02)	0.28 (0.02)	0.27 (0.02)				
	F	0.26 (0.03)	0.26 (0.02)	0.26 (0.03)				

Stride length (m)	S	1.61 (0.18)	1.60 (0.21)	1.67 (0.26)	0.562	**<0.001** ^*∗*^	0.784	S < P, F; P < F
	P	1.77 (0.18)	1.77 (0.24)	1.81 (0.26)				
	F	1.93 (0.21)	1.91 (0.25)	1.97 (0.27)				

Ankle dorsiflexion at touchdown (°)	S	5.98 (10.47)	2.76 (2.35)	3.75 (4.92)	0.336	0.263	0.553	—
	P	5.56 (10.21)	2.74 (2.38)	4.08 (3.80)				
	F	6.30 (10.49)	2.91 (2.66)	4.45 (3.75)				

Ankle inversion at touchdown (°)	S	1.95 (2.11)	1.97 (2.18)	2.24 (2.13)	0.617	**0.003** ^*∗*^	0.234	S > F
	P	2.06 (1.75)	1.23 (2.65)	1.93 (2.10)				
	F	1.52 (2.03)	1.93 (2.10)	1.55 (2.04)				

Ankle sagittal RoM (°)	S	29.61 (3.84)	29.77 (3.32)	29.76 (2.86)	0.864	**<0.001** ^*∗*^	0.771	S < P, F
	P	30.63 (3.64)	31.01 (4.57)	30.65 (3.15)				
	F	31.18 (3.37)	31.40 (3.86)	31.91 (3.12)				

Ankle frontal RoM (°)	S	9.60 (2.56)	8.64 (2.00)	9.36 (2.27)	0.534	**<0.001** ^*∗*^	0.336	F > S, P
	P	9.68 (2.85)	9.59 (2.47)	9.75 (2.03)				
	F	10.60 (2.77)	9.88 (2.95)	10.53 (2.68)				

S, slow; P, preferred, and F, fast. ^*∗*^Indicating a significant effect, *P* < 0.05. BW, bodyweight.

The article "Effectiveness of Insole Colour on Impact Loading and Lower-Limb Kinematics When Running at Preferred and Nonpreferred Speeds" was published in 2021. Journal: J Healthc Eng.

**Table 2:** Coefficient of variation (CV) of ground reaction force and spatiotemporal and joint angle variables by insole colour and speed conditions.

Variables	Speed	Red	Blue	White	ANOVA (*P* value)			Post hoc
					Colour	Speed	Interaction	
Peak impact force (%)	S	2.91 (1.26)	2.92 (0.92)	2.80 (1.08)	0.895	0.420	0.134	
	P	2.20 (0.89)	2.57 (0.78)	2.94 (1.46)				
	F	3.25 (2.58)	2.49 (0.89)	2.48 (0.71)				

Max loading rate (%)	S	14.26 (4.20)	11.74 (4.56)	14.13 (5.06)	**0.033** ^*∗*^	0.393	0.817	Red > blue
	P	14.70 (5.82)	11.98 (5.16)	13.18 (3.89)				
	F	13.27 (5.34)	11.83 (3.90)	11.99 (3.18)				

Contact time (%)	S	3.26 (1.63)	3.04 (1.27)	3.02 (2.28)	0.697	0.061	0.460	—
	P	2.75 (0.85)	2.37 (1.24)	2.76 (0.82)				
	F	2.81 (0.92)	2.97 (1.64)	2.41 (0.88)				

Stride length (%)	S	1.64 (0.68)	1.36 (0.57)	1.44 (0.73)	0.780	0.861	0.254	—
	P	1.37 (0.37)	1.37 (0.59)	1.71 (0.84)				
	F	1.58 (1.41)	1.48 (0.60)	1.19 (0.43)				

Ankle dorsiflexion at touchdown (%)	S	7.89 (3.38)	10.47 (5.44)	9.32 (4.75)	0.208	0.652	0.959	—
	P	8.87 (3.14)	8.85 (5.12)	8.50 (4.55)				
	F	8.94 (6.65)	7.38 (2.65)	10.00 (5.55)				

Ankle inversion at touchdown (%)	S	55.00 (17.28)	109.19 (122.31)	64.67 (75.11)	0.570	0.108	0.446	—
	P	52.83 (23.10)	67.42 (60.17)	56.96 (32.80)				
	F	68.62 (43.70)	105.76 (134.26)	135.91 (226.86)				

Ankle sagittal RoM (%)	S	9.47 (3.36)	7.40 (2.77)	7.32 (3.50)	0.182	**0.038** ^*∗*^	0.144	S > P, F
	P	7.01 (2.37)	6.82 (2.39)	6.83 (3.16)				
	F	7.03 (1.66)	8.09 (3.41)	6.23 (2.64)				

Ankle frontal RoM (%)	S	16.54 (4.84)	18.51 (6.82)	18.13 (7.76)	0.643	0.356	0.508	—
	P	17.64 (7.31)	17.84 (8.39)	17.42 (6.07)				
	F	17.51 (5.29)	17.48 (12.03)	14.41 (4.11)				

S, slow; P, preferred; F, fast. ^*∗*^Indicating a significant effect, *P* < 0.05.

## Data Availability

The data are available upon reasonable request.

## References

[1] van Gent R. N., Siem D., van Middelkoop M. (2007). Incidence and determinants of lower extremity running injuries in long distance runners: a systematic review ∗ COMMENTARY. *British Journal of Sports Medicine*.

[2] Hardin E. C., Hamill J. (2002). The influence of midsole cushioning on mechanical and hematological responses during a prolonged downhill run. *Research Quarterly for Exercise & Sport*.

[3] Law J. C. L., Wong T. W. L., Chan D. C. L., Lam W.-K. (2018). Effects of shoe top visual patterns on shoe wearers’ width perception and dynamic stability. *Perceptual & Motor Skills*.

[4] Sun X., Lam W. K., Zhang X., Wang J., Fu W. (2020). Systematic review of the role of footwear constructions in running biomechanics: implications for running-related injury and performance. *Journal of Sports Science & Medicine*.

The article "Effectiveness of Insole Colour on Impact Loading and Lower-Limb Kinematics When Running at Preferred and Nonpreferred Speeds" was published in 2021. Journal: J Healthc Eng.

[5] Lucas-Cuevas A. G., Pérez-Soriano P., Priego-Quesada J. I., Llana-Belloch S. (2014). Influence of foot orthosis customisation on perceived comfort during running. *Ergonomics*.

[6] O’Leary K., Vorpahl K. A., Heiderscheit B. (2008). Effect of cushioned insoles on impact forces during running. *Journal of the American Podiatric Medical Association*.

[7] Lam W. K., Lee W. C., Ng S. O., Zheng Y. (2019). Effects of foot orthoses on dynamic balance and basketball free-throw accuracy before and after physical fatigue. *Journal of Biomechanics*.

[8] Lam W.-K., Pak L.-Y., Wong C. K.-W. (2020). Effects of arch-support orthoses on ground reaction forces and lower extremity kinematics related to running at various inclinations. *Journal of Sports Sciences*.

[9] Spooner S., Griffiths I. (2021). Should colour be considered as a significant design variable in foot orthoses prescription writing?. *Preprints*.

[10] Elliot A. J., Maier M. A. (2014). Color psychology: effects of perceiving color on psychological functioning in humans. *Annual Review of Psychology*.

[11] Hill R. A., Barton R. A. (2005). Red enhances human performance in contests. *Nature*.

[12] Wiercioch-Kuzianik K., Bąbel P. (2019). Color hurts. The effect of color on pain perception. *Pain Medicine*.

[13] Wylde V., Wells V., Dixon S., Gooberman-Hill R. (2014). The colour of pain: can patients use colour to describe osteoarthritis pain?. *Musculoskeletal Care*.

[14] Elliot A. J., Aarts H. (2011). Perception of the color red enhances the force and velocity of motor output. *Emotion*.

[15] García-Rubio M. A., Picazo-Tadeo A. J., González-Gómez F. (2011). Does a red shirt improve sporting performance? Evidence from Spanish football. *Applied Economics Letters*.

[16] Piatti M., Savage D. A., Torgler B. (2012). The red mist? Red shirts, success and team sports. *Sport in Society*.

[17] Rowe C., Harris J. M., Roberts S. C. (2005). Sporting contests - seeing red? Putting sportswear in context. *Nature*.

[18] Kam K. K. W., Uiga L., Lam W. K., Capio C. M. (2021). The colour we wear: impact on self-predicted and actual motor performance. *Journal of Sport & Exercise Science*.

[19] Dreiskaemper D., Strauss B., Hagemann N., Büsch D. (2013). Influence of red Jersey color on physical parameters in combat sports. *Journal of Sport & Exercise Psychology*.

[20] Wang Y., Lam W. K., Cheung C. H., Leung A. K. L. (2020). Effect of red arch-support insoles on subjective comfort and movement biomechanics in various landing heights. *International Journal of Environmental Research and Public Health*.

The article "Effectiveness of Insole Colour on Impact Loading and Lower-Limb Kinematics When Running at Preferred and Nonpreferred Speeds" was published in 2021. Journal: J Healthc Eng.

[21] Zunker C., Karr T. M., Sherman R. T. Perceptions of running performance: the role of clothing fit. *The Sport Journal*.

[22] Tartaruga M. P., Brisswalter J., Peyré-Tartaruga L. A. (2012). The relationship between running economy and biomechanical variables in distance runners. *Research Quarterly for Exercise & Sport*.

[23] Mercer J. A., Vance J., Hreljac A., Hamill J. (2012). Relationship between shock attenuation and stride length during running at different velocities. *European Journal of Applied Physiology*.

[24] Abernethy B., Hanna A., Plooy A. (2002). The attentional demands of preferred and non-preferred gait patterns. *Gait & Posture*.

[25] Cavanagh P. R., Rodgers M. M. (1987). The arch index: a useful measure from footprints. *Journal of Biomechanics*.

[26] Marey H. M., Semary N. A., Mandour S. S. (2014). Ishihara electronic color blindness test: an evaluation study. *Ophthalmology Research: International Journal*.

[27] Gottschall J. S., Kram R. (2005). Ground reaction forces during downhill and uphill running. *Journal of Biomechanics*.

[28] Wang Y., Lam W. K., Wong C. K., Park L. Y., Tan M. F., Leung A. K. L. (2020). Effectiveness and reliability of foot orthoses on impact loading and lower limb kinematics when running at preferred and nonpreferred speeds. *Journal of Applied Biomechanics*.

[29] Cohen J. (2013). *Statistical Power Analysis for the Behavioral Sciences*.

[30] Pohl M. B., Hamill J., Davis I. S. (2009). Biomechanical and anatomic factors associated with a history of plantar fasciitis in female runners. *Clinical Journal of Sport Medicine*.

[31] Wang X., Ma Y., Hou B. Y., Lam W. K. (2017). Influence of gait speeds on contact forces of lower limbs. *Journal of Healthcare Engineering*.

[32] Orendurff M. S., Kobayashi T., Tulchin-Francis K. (2018). A little bit faster: lower extremity joint kinematics and kinetics as recreational runners achieve faster speeds. *Journal of Biomechanics*.

[33] Greenlees I., Leyland A., Thelwell R., Filby W. (2008). Soccer penalty takers’ uniform colour and pre-penalty kick gaze affect the impressions formed of them by opposing goalkeepers. *Journal of Sports Sciences*.

[34] Attrill M. J., Gresty K. A., Hill R. A., Barton R. A. (2008). Red shirt colour is associated with long-term team success in English football. *Journal of Sports Sciences*.

[35] Roberts J., Jones R., Harwood C., Mitchell S., Rothberg S. (2001). Human perceptions of sports equipment under playing conditions. *Journal of Sports Sciences*.

[36] Van Emmerik R. E. A., Miller R. H., Hamill J. (2014). Dynamical systems analysis of coordination. *Human Kinetics*.

The article "Effectiveness of Insole Colour on Impact Loading and Lower-Limb Kinematics When Running at Preferred and Nonpreferred Speeds" was published in 2021. Journal: J Healthc Eng.

[37] Kinchington M. A., Ball K. A., Naughton G. (2011). Effects of footwear on comfort and injury in professional rugby league. *Journal of Sports Sciences*.

[38] Luo G., Stergiou P., Worobets J., Nigg B., Stefanyshyn D. (2009). Improved footwear comfort reduces oxygen consumption during running. *Footwear Science*.

[39] Mills K., Blanch P., Chapman A. R., McPoil T. G., Vicenzino B. (2010). Foot orthoses and gait: a systematic review and meta-analysis of literature pertaining to potential mechanisms. *British Journal of Sports Medicine*.

